This article has been retracted.

# Prediction of Ovarian Cancer Response to Therapy Based on Deep Learning Analysis of Histopathology Images

**DOI:** 10.3390/cancers15164044

**Published:** 2023-08-10

**Authors:** Yuexin Liu, Barrett C. Lawson, Xuelin Huang, Bradley M. Broom, John N. Weinstein

**Affiliations:** 1 Department of Bioinformatics and Computational Biology, The University of Texas MD Anderson Cancer Center, Houston, TX 77030, USA; bmbroom@mdanderson.org; 2 Department of Pathology, The University of Texas MD Anderson Cancer Center, Houston, TX 77030, USA; bclawson@mdanderson.org; 3 Department of Biostatistics, The University of Texas MD Anderson Cancer Center, Houston, TX 77030, USA; xlhuang@mdanderson.org; 4 Department of Systems Biology, The University of Texas MD Anderson Cancer Center, Houston, TX 77030, USA

**Keywords:** deep learning, neural network, chemotherapy response, occlusion sensitivity analysis, Inception V3, convolutional neural network, spatialomic, spatialomics, platinum chemotherapy, histopathology, ovarian cancer, artificial intelligence

## Abstract

**Simple Summary:**

Ovarian cancer remains the leading cause of mortality from gynecologic cancer. In this study, we present a deep-learning artificial intelligence framework that uses pre-treatment histopathology images of high-grade ovarian cancers to predict the cancer’s sensitivity or resistance to subsequent platinum-based chemotherapy. Analyses of this type could provide fast, inexpensive prediction of response to therapy at the time of initial pathological diagnosis.

**Abstract:**

Background: Ovarian cancer remains the leading gynecological cause of cancer mortality. Predicting the sensitivity of ovarian cancer to chemotherapy at the time of pathological diagnosis is a goal of precision medicine research that we have addressed in this study using a novel deep-learning neural network framework to analyze the histopathological images. Methods: We have developed a method based on the Inception V3 deep learning algorithm that complements other methods for predicting response to standard platinum-based therapy of the disease. For the study, we used histopathological H&E images (pre-treatment) of high-grade serous carcinoma from The Cancer Genome Atlas (TCGA) Genomic Data Commons portal to train the Inception V3 convolutional neural network system to predict whether cancers had independently been labeled as sensitive or resistant to subsequent platinum-based chemotherapy. The trained model was then tested using data from patients left out of the training process. We used receiver operating characteristic (ROC) and confusion matrix analyses to evaluate model performance and Kaplan–Meier survival analysis to correlate the predicted probability of resistance with patient outcome. Finally, occlusion sensitivity analysis was piloted as a start toward correlating histopathological features with a response. Results: The study dataset consisted of 248 patients with stage 2 to 4 serous ovarian cancer. For a held-out test set of forty patients, the trained deep learning network model distinguished sensitive from resistant cancers with an area under the curve (AUC) of 0.846 ± 0.009 (SE). The probability of resistance calculated from the deep-learning network was also significantly correlated with patient survival and progression-free survival. In confusion matrix analysis, the network classifier achieved an overall predictive accuracy of 85% with a sensitivity of 73% and specificity of 90% for this cohort based on the Youden-J cut-off. Stage, grade, and patient age were not statistically significant for this cohort size. Occlusion sensitivity analysis suggested histopathological features learned by the network that may be associated with sensitivity or resistance to the chemotherapy, but multiple marker studies will be necessary to follow up on those preliminary results. Conclusions: This type of analysis has the potential, if further developed, to improve the prediction of response to therapy of high-grade serous ovarian cancer and perhaps be useful as a factor in deciding between platinum-based and other therapies. More broadly, it may increase our understanding of the histopathological variables that predict response and may be adaptable to other cancer types and imaging modalities.

## 1. Introduction

Ovarian carcinoma (OvCa) remains the leading cause of mortality from gynecologic cancer, with estimated 21,410 new cases and 13,770 deaths in the United States alone in 2021 [1]. A standard treatment protocol for advanced-stage epithelial OvCa includes cytoreductive surgery followed by platinum-based combination chemotherapy. However, the majority of patients eventually relapse with a generally incurable disease, mainly due to the emergence of resistance to chemotherapy [2,3]. Chemotherapy imposes significant toxicity and cost [4]; hence, early identification of patients whose cancers are resistant to chemotherapy is a goal of precision medicine.

OvCa patients with *BRCA1/2* mutations (germline or somatic) respond better to platinum-based treatment and have substantially longer survival than non-carriers [5], and additional genomic markers of response have been identified. For example, we previously found that mutations in members of the ADAMTS (a disintegrin and metalloproteinase with thrombospondin motifs) gene family were significantly associated with an improved response to platinum-based chemotherapy and substantially longer survival in OvCa patients, independent of *BRCA1/2* mutation [6]. The association of ADAMTS mutations with drug sensitization in ovarian cancer cells was functionally validated using ovarian cancer in vitro and in vivo model systems [7]. However, additional predictors of response would be useful.

In addition to genomic aberrations, morphological alterations have long been a hallmark of cancer pathology. Morphologic features can be correlated with cellular functions such as cell growth, apoptosis, differentiation, and migration [8,9,10] and are routinely used for cancer diagnosis in clinical practice. Genetic testing for *BRCA1/2* mutations is currently performed in clinical practice on ovarian cancer patients to predict drug sensitivity. However, only 15–20% of the cancers have a *BRCA1/2* mutation (germline or somatic) [6], and therefore response to chemotherapy in the remaining percentage of patients with ovarian cancer is not subject to prediction on the basis of that genomic marker.

Convolutional neural networks (CNNs) consisting of convolution, activation, and pooling layers represent a specific type of deep learning architecture that is well suited to image analysis tasks [11]. The development of graphics processing units (GPUs), the accessibility of large amounts of data, and the high accuracies achievable have caused a surge in the application of deep learning to image analysis in the last few years [12,13]. Several CNNs have been successfully designed for automated detection, segmentation, or classification of medical and whole-slide histopathological images for a wide array of cancer types [11,14,15,16,17]. Computational pathology using deep learning techniques may lead to quick, inexpensive methods for characterizing the tumor microenvironment [18,19,20,21], distinguishing tumor subtypes, correctly grading tumors, and predicting gene mutations based on histopathology images [22,23,24,25]. Such analysis methods can, in principle, be applied to all types of what we might term ‘spatialomic’ technologies, including those based on sequencing and multiplexed labeling with antibodies. For ovarian cancers, Wu et al. have used a deep learning model and hematoxylin–eosin (H&E) stained tissue sections to classify ovarian cancer histologic subtypes automatically [26], and Shin et al. leveraged an image set obtained from The Cancer Image Archive (TCIA) to distinguish malignant tissues from normal background based on a CNN model [27]. Wang et al. [28] developed a weakly supervised deep learning approach to predict the therapeutic response of ovarian cancers to bevacizumab based on histopathology images, and a similar weakly-supervised neural network was proposed to discriminate ovarian cancer patients with extremely different platinum-free intervals. The patient cohort used in that study was relatively small, and a majority of ovarian cancer patients with platinum-free intervals in between the two extremes remained undetermined [29]. Yu et al. employed a series network architecture (VGGNet) with regression output to predict platinum-free intervals of ovarian cancer patients from histopathology images [30]. Thus far, no similar studies have used deep learning network algorithms and histopathology images to classify ovarian cancer patients into resistant or sensitive categories in a large patient population [31]. 

Using whole-slide H&E-stained ovarian tumor samples from The Cancer Genome Atlas (TCGA), we previously applied a hand-crafted image segmentation, feature-based machine learning approach to identify morphologic features associated with chemotherapy response in OvCa patients [32]. In the present study, we have taken a different approach, using a deep learning neural network method based on the Inception V3 directed acyclic graph architecture [33] to predict chemotherapy response status using the same image set as in our previous image segmentation approach [32]. In addition, we piloted occlusion sensitivity analysis (OSA) to identify morphological features in the pathology images that are associated with resistance to chemotherapy. This proof-of-principle study suggests that deep learning, in particular with the Inception V3 architecture, can be applied to other cancer types and probably, with modifications, to other imaging modalities.

## 2. Methods

### 2.1. TCGA Ovarian Cancer Whole-Slide Image Dataset 

Whole-slide, frozen-section, H&E-stained images of ovarian cancer analyzed in this study (all of them designated as high-grade serous carcinoma) were downloaded from the TCGA Genomic Data Commons portal. Platinum responsiveness labels (sensitive/resistant) of the cancers provided by the TCGA database [34] were used as our ground truth in the analysis. The cancers were categorized as platinum-resistant if the platinum-free interval was less than 6 months and the patient experienced progression or recurrence. They were categorized as platinum-sensitive if the platinum-free interval was 6 months or more without evidence of progression or recurrence. The entire cohort consisted of 174 chemotherapy-sensitive (chemo-sensitive) patients and 74 chemotherapy-resistant (chemo-resistant) patients (**Table 1**). The average age of the cohort was 60.0 years (range, 30.5 to 87.5). The majority of the patients were defined as WHO high grade (grade 3) with stage III or IV disease, and 37 were defined as “grade 2”. To assess whether the relationship between tumor grade and chemotherapy response was more than expected by chance, we created a contingency table and performed Fisher’s exact test. The results did not demonstrate a statistically significant association of chemotherapy resistance with tumor grade (*p* = 0.3287) (**Supplementary Table S1**), tumor stage (*p* = 0.216, Fisher’s exact test) (**Supplementary Table S2**), or patient age (*p* = 0.087, Mann–Whitney test) (**Supplementary Figure S1**). 

### 2.2. Tile Datastore Generation via Image Preprocessing

Based on high-resolution images, regions of interest (ROIs) at a magnification of 20X (size: 1072 × 648 pixels) were selected by an expert gynecologic pathologist using the Aperio ImageScope (Leica Biosystems) [32]. That selection was performed to ensure that the majority of the fields to be analyzed represented tumor. We know of no reason to expect that choice of ROIs would introduce significant bias, although that possibility cannot be ruled out. To account for spatial heterogeneity of the tumor tissues, an average of 10 ROIs per slide from different views of the tissue blocks were selected from the H&E-stained ScanScope virtual slide set (**Supplementary Figure S2**). As a result, a total of 2389 ROIs were selected, 1680 of them from sensitive tumors and 709 from resistant ones. ROIs were further tiled in non-overlapping 299 × 299-pixel windows, and incomplete tiles smaller than the window size were excluded. That process generated over 14,000 tiles in total for image analysis. For detailed information regarding the number of tiles, ROIs, and slides for resistant/sensitive classification, see **Supplementary Table S3**.

### 2.3. Deep Learning with Convolutional Neural Network

For independent testing of models generated, we left a total of 40 slides (2370 tiles) out of the training process. We then used 95% of the remaining tiles for training and 5% of the tiles for validation (**Supplementary Table S3**). Only the training tiles (but not the validation or test tiles) were used to update network parameters. The validation tiles were used to evaluate network performance during the training process. The test-set tiles were then used to assess the network generalizability after the network had been fully trained. To ensure the reproducibility of the results, the training and test process was repeated a total of 16 times after creating random splits of the training and validation datasets with a ratio of 95:5 while retaining the same test set. To assess the effect of class imbalance on the results, we performed two different experiments. One was to upsize the number of resistance images; the other was to downsize the number of sensitive images so that the numbers of resistant and sensitive images were matched with each other. We based our CNN model on the Inception V3 architecture developed by Google researchers [33]. That architecture makes use of inception modules that include multiple convolutions with different filter sizes and a max or average pooling layer. The Inception V3 architecture starts with five convolutional and two max pooling layers that are then followed by eleven inception modules. The architecture ends the sequence with an average pooling layer, a dropout layer, a fully connected layer, and then a softmax output layer. For drug response classification, we trained the whole network, including the last fully connected layer and also the prior layers.

### 2.4. Training the Inception V3 Network

We trained the Inception V3 architecture following the procedure previously described [33]. The network parameters were first initialized to those that were achieved by ImageNet competition and then updated on our training set data via backpropagation. We used RMSProp optimization, with a learning rate of 10^−5^, gradient decay factor of 0.99, regularization of 10^−4^, and epsilon of 10^−8^ for training the weights. In addition to the fully connected layer, we also optimized the weights and biases of all previous learnable layers (i.e., the convolution and activation layers). That strategy was used for the classification of drug response. The training jobs were run for 50 epochs, which corresponded to over 50,000 iterations. We computed the predictive accuracy on the training and validation datasets, and similar to other studies [24,25], we used the model with the best validation score as our final model for application to the test set, which had been left out of the entire training process. 

### 2.5. Statistical Analysis

Once the training phase was completed, we then used the test dataset (composed of tiles not used in training) to evaluate model performance. The probabilities for each slide were aggregated using the mean probability of its tiles. ROC curves and the corresponding AUCs were computed [35] using Matlab and GraphPad 9.0 software. Confusion matrix charts were computed and visualized using Matlab, and an optimal cut-point (derived from the ROC curve) was calculated by the Youden J-index method [36]. Slide probability distributions and relationships to chemotherapy response in the same test dataset were analyzed using the two-tailed Mann–Whitney U-test. 

We used the Kaplan–Meier method [37] to examine the association between the predicted slide probabilities and patient survival [6,34], including both overall survival (OS) and progression-free survival (PFS). The patients were then dichotomized into two groups based on the predicted slide probabilities with the Youden J-index cutoff (0.2612 in this case) [36]. Survival differences between the two groups were assessed using the log-rank test. In the multivariate Cox proportional hazards model analysis, the slide probability score, stage, and tumor grade were treated as ordinal categorical variables, and patient age was treated as a continuous variable. The Wald test was used to evaluate survival differences in the multivariate analysis.

### 2.6. Identification of Histopathologic Features Associated with Chemotherapy Response

In an attempt to identify histopathological factors that might explain the predictiveness of the neural network results, we piloted the use of occlusion sensitivity analysis (OSA) [38]. In OSA, the network’s sensitivity to serial perturbations of small regions of the image is determined. The mask size used was 15 × 15 pixels, and the mask value was defined as the channel-wise mean of the input data. The mask was moved across the image, and the change in probability score for the given class was determined as a function of mask position. The step size for traversing the mask across the image was 10 pixels in both vertical and horizontal directions. Finally, we used bicubic interpolation to produce a smooth map the same size as the input data. The occlusion sensitivity map highlights which parts of the image are most important to the classification. That is, when that part of the image is occluded, the probability score for the predicted class rises or falls accordingly. By convention, red areas of the map have a higher positive value and are evidence for the given class. When red areas are occluded, the probability score for the class probability, as predicted by the deep learning algorithm, decreases. Blue areas of the map with small positive values or negative values indicate parts of the image that lead to negligible change or opposite change in the score when occluded, suggesting that their features have negligible or opposite impact on the predicted class. To identify the features more clearly, we superimposed the OSA maps on the original tile images or else toggled back and forth between the map and the corresponding histopathology tile. 

## 3. Results

### 3.1. A Deep Learning Framework for Digital Analysis of Histopathology Images 

In this study, we sought to develop a deep learning framework for automatic predictive analysis of tumor slides using whole-slide images publicly available in TCGA’s Cancer Digital Image Archive (CDIA). Our overall computational strategy is summarized in **Figure 1**. We first downloaded H&E-stained whole-slide images from the TCGA CDIA (**Figure 1****a**). Because many of the slide images included non-tumor areas, regions of interest (ROIs) were then manually selected at 20x magnification by a gynecologic pathologist (**Figure 1**a). Because the ROIs were much larger than the input size usable by the neural network, we trained, validated, and tested the network using 299 × 299-pixel tiles obtained from non-overlapping ‘patches’ of the ROIs (**Figure 1****a**). The tiles (six per ROI) were labeled as chemo-sensitive or chemo-resistant (i.e., as having been obtained from chemo-sensitive or chemo-resistant patients), and a tile datastore was generated (**Figure 1****a**). The tiles were further split into training, validation, and test sets (**Figure 1****b**). The training and validation tiles were used to train the Inception V3 network architecture, as described in the Methods section, and to select the final model (**Figure 1****c**). Tiles in the independent test set were then used to evaluate model performance after aggregation of tiles to the slide (i.e., patient) level once the fully trained neural network had been obtained (**Figure 1****d**). Aggregation to the patient level was appropriate because that was the level of pre-labeled sensitivity or resistance.

### 3.2. Testing and Tile Aggregation Pipeline

Once the training phase was completed, we tested the fully trained model with the test dataset (**Figure 2**). Tiles generated from the test slides (**Figure 2****a**) were used as inputs and fed into the trained deep learning model (**Figure 2****b**), which then generated the class probability (range 0 to 1) for each tile (**Figure 2****c**). We then aggregated the per-tile classification results on an ROI basis by averaging the probabilities obtained for the six tiles from the ROI (**Figure 2****d**). Similarly, we further aggregated the per-ROI classification results on a slide basis by averaging the probabilities obtained on the ROIs from the same slide (**Figure 2****e**). For each slide, we then obtained the class probability at the slide (i.e., patient) level, from which we calculated the AUC statistics (**Figure 2****f**).

### 3.3. The Deep Learning Model Predicts Chemotherapy Response from Ovarian Histopathology Images

Next, we tested the generalization error of the deep learning model with a test set comprised of 29 chemo-sensitive and 11 chemo-resistant cancers. After aggregation of the statistics on a slide (i.e., patient) basis, violin plot and ROC curve analysis (**Figure 3****a,b**) showed that chemotherapy response could be predicted using our deep-learning approach, which yielded a Cohen’s d of 1.33 (considered “large”) and an AUC value of 0.843. Next, we applied the Youden J index and constructed the confusion matrix (**Figure 3****c**). The predicted classes obtained by the Inception V3 deep learning algorithm were significantly associated with the true class (*p* = 0.003, Fisher’s exact test). This result contrasts with the non-significant association of chemotherapy response with clinical factors (i.e., grade, stage, age) in the same cohort (see Methods for direct comparison). Approximately 85% of patients were correctly classified in terms of drug sensitivity on the basis of pre-treatment histopathology, with a sensitivity of 73% and a specificity of 90% at the Youden J point (**Figure 3****c**). The large value of Cohen’s d (1.33) indicates that the difference between sensitive and resistant may be “meaningful” as well as statistically significant. Repeated random sub-sampling to obtain 16 different training sets gave an average test set AUC value of 0.846 ± 0.009 (SE) (range, 0.781–0.900) (**Figure 3****d**), consistent with the result for the first random choice of the training set. Calculations using upsizing and downsizing to match sensitive and resistant dataset sizes indicated that the AUC results were not much impacted by class imbalance (**Supplementary Figure S3**).

We next determined the relationship between predicted probabilities from the slides and patient outcome, including both overall survival (OS) and progression-free survival (PFS). When the Youden J-index-based cut point was applied, Kaplan–Meier analysis showed that the network classifier correlated significantly with both OS (**Figure 4****a**, *p* = 0.0084) and PFS (**Figure 4****b**, *p* = 0.0226). To test whether that result was independent of known predictive variables such as stage, grade, or age, we performed multivariate analysis using the Cox proportional hazards model with the network classifier and the other variables as covariates. After adjustment for stage, grade, and age, the Inception V3 probability score correlated with OS (*p* = 0.013) and PFS (*p* = 0.045) (**Supplementary Tables S4 and S5**). Those results further confirmed the prediction of chemotherapy response using the Inception V3 deep learning model.

### 3.4. Visualization of Chemotherapy Response-Associated Features Identified by the Deep Learning Model

To assist pathologists in their classification of whole-slide images of ovarian cancer tissues, we next sought to identify morphological features associated with chemotherapy response by using OSA (**Figure 5**). For high-confidence tiles (**Figure 5****a**), the dynamic range of the occlusion sensitivity map is narrow, and the blue areas denote smaller positive values (**Figure 5****b**). The overlaid image (**Figure 5****c**) explicitly shows features associated with responsive disease. More instructive are tiles for which the network is ambivalent about the prediction (i.e., with a probability equal to ~0.5 for resistant and ~0.5 for sensitive) (**Figure 5****d**). In such cases, the occlusion sensitivity map has a much wider dynamic range and can be used to compare which features (e.g., cell types) in the image the network identified with different response classes (**Figure 5****e**). From the overlaid image (**Figure 5****f**), we could discern features or regions that contributed to the chemotherapy resistance (red areas with positive values). In contrast, blue areas of the map with negative values are parts of the image that lead to an increase in the score when occluded. Often those areas are suggestive of the opposite class (“sensitive” in this case).

## 4. Discussion

This study demonstrates the use of an Inception V3 convolution neural network deep learning model to predict the response of high-grade serous ovarian cancer patients to platinum-based chemotherapy on the basis of pre-treatment histopathology slides. The deep learning classifier achieved a mean ROC AUC of 0.846 ± 0.009 with an accuracy of 85% in correctly classifying tumors previously labeled as resistant or sensitive in the TCGA ovarian cancer dataset. Accordingly, the predictions also correlated with OS and PFS. Those studies demonstrated that features learned by the deep learning model can distinguish resistant from sensitive diseases despite staining and processing artifacts present in the TCGA frozen sections. Occlusion sensitivity analysis (OSA) [38] could further assist in the prediction of chemotherapy response at the time of pathological diagnosis, but further studies, including multiplexed immunohistochemical analyses, will be necessary for a fuller interpretation of the factors involved.

We previously reported that particular nucleus morphology features (size and shape) in segmented histopathology images were correlated with chemotherapy response in the same ovarian cancer samples as those used in the present study [32]. Different from that “feature engineering” approach to prediction, which requires the definition of problem-specific features [32], deep learning networks learn image feature representations from the data autonomously. As a result, the need for domain knowledge to achieve useful results is greatly decreased [39]. Deep learning image analysis networks are trained end-to-end directly from image labels and raw pixels; hence, they show potential for general and highly variable tasks across many fine-grained object categories. Generalizability of this study’s results is suggested by qualitatively consistent data obtained in an independent study [30] using a different (series-structured) deep learning architecture (VGGNet), slide tiling strategy, composition of cohort, and factor analysis methodology in generating and analyzing a regression model for prediction of the response to therapy.

Deep learning models are often described as “black-box” due to the opaque nature of the algorithms, which are trained rather than explicitly programmed; hence, reasons for results are difficult for humans to interpret. Our introduction of OSA [38] is an initial attempt to ameliorate that uncertainty by discovering what parts of an image are most important for deep learning classification.

This study has limitations. (i) The sizes of the overall cohort (248 patients) and test set (40 patients) were relatively small. However, that was easily sufficient to achieve statistically robust results for the two-class prediction; (ii) There was no independent patient cohort from a source other than TCGA to evaluate the model for generalization of results. However, it should be noted that the TCGA samples were obtained from numerous institutions and represent a wide spread of age, stage, processing methods, and other non-histopathological variables. (iii) The dataset comprises only high-grade serous carcinomas and predominantly advanced-stage tumors that do not fully represent the diversity and clinical heterogeneity of ovarian cancers. Of note, the TCGA dataset includes “grade 2” for high-grade serous carcinoma. That is not a currently recognized grade for ovarian serous tumors, which are now defined just as low- or high-grade serous; however, no significant difference in response was noted in this study that would indicate a large difference between the “grade 2” and “grade 3” tumors. (iv) This study used only ROIs and included pre-treatment samples only from patients who later received frontline platinum-based chemotherapy. (v) The TCGA specimens analyzed were frozen sections, adding artifacts beyond those that would be seen with H&E slides prepared from formalin-fixed paraffin-embedded (FFPE) tissues. Hence, more accurate predictions of response to therapy might be obtainable by the CNN system from FFPE samples. Whereas FFPE slides are less than ideal for sequencing studies, they are much better than frozen in terms of visual features as well as availability in pathology archives. Further evaluation of the CNN classifier for a larger cohort, FFPE slides, and/or tissue microarrays would provide additional useful information. However, the CNN framework presented here could potentially add to the corpus of information on clinical trial patients as they are selected for platinum-based or more recently developed therapeutic regimens.

## 5. Conclusions

This is a proof-of-principle study demonstrating the application of an Inception V3 deep learning model for prediction of ovarian cancer response to platinum-based chemotherapy based solely on histopathology images. Its results, if further developed, and if combined with other predictive variables (e.g., including nucleus morphology, demographic data, stage, grade, and ‘omic’ [40] profilingmay have utility in clinical management. The desirability of extending the approach to FFPE samples and additional tumor types is apparent.

## Figures and Tables

**Figure 1:** **Computational pipeline for training and testing the deep learning model.** (**a**), A tile datastore was generated from images of ovarian cancer tissues. (**b**), Tiles were then separated into training, validation, and held-out test sets. (**c**), The Inception V3 architecture was fully trained using the training and validation tiles. (**d**), Testing was performed on tiles from the test set and then aggregated per slide (i.e., per patient) to extract the ROC statistics.

**Figure 2:** **Testing and tile aggregation pipeline.** (**a**), Tiles from test slides. (**b**), The trained deep learning network. (**c**), The predicted probabilities for all the tiles. (**d**), Tile aggregation per ROI. (**e**), ROI aggregation per slide. (**f**), Class prediction on the basis of slide probability.

**Figure 3:** **Classification of chemotherapy response status on a test set of 40 ovarian cancer patients**. (**a**), Distribution of predicted slide probabilities of chemotherapy response (i.e., resistant or sensitive) with slide probability calculated after tile aggregation. (**b**), Receiver operating characteristic (ROC) curve from the first random test set of 40 slides. (**c**), Illustrative confusion matrix for the test set. (**d**), Test-set receiver operating characteristic (ROC) curves for 16 random training set samplings.

**Figure 4:** Association of the slide probabilities with patient overall survival (**a**) and progression-free survival (**b**). Note that this result is not independent of optimization through selection of the Youden J-index cut point.

**Figure 5:** Visualization of chemotherapy-response-associated features in representative tile images identified by the deep learning model. (**a**), A high-confidence tile image predicted by the deep learning network to be from a sensitive tumor with a probability score of 0.98. (**b**), Occlusion sensitivity analysis (OSA) map for the sensitive class. (**c**), Image superimposing the OSA map on the original tile image. (**d**), An ambiguous tile image predicted to have essentially identical scores for sensitivity and resistance. (**e**), OSA map for the resistant class for (**d**). (**f**), Image superimposing the OSA map on the original tile image (**d**).

**Table 1:** Clinicopathologic characteristics of TCGA patients with serous OvCa in the cohort used for training, validating, and testing the convolutional neural network system.

No. of Patients	248		
Chemotherapy response ^ξ^			
Resistant		74	
Sensitive		174	
Age			
Mean, years [SD]	60.0 [11.4]		
Range	30.5–87.5		
FIGO Stage ^¶^			
II	13		
III	196		
IV	36		
Unknown	3		
WHO Grade			
2	37		
3	204		
Unknown	7		
Vital status			
Alive	94		
Dead	150		
Unknown	4		
Recurrent disease ^ζ^			
Yes	216		
No	29		
Unknown	3		

Abbreviations: TCGA, The Cancer Genome Atlas; FIGO, International Federation of Gynecology and Obstetrics; SD, standard deviation; WHO, World Health Organization. ^ξ^: Platinum status was defined as resistant if the platinum-free interval was less than 6 months and the patient experienced progression or recurrence. It was defined as sensitive if the platinum-free interval was 6 months or more and there was no evidence of progression or recurrence. ^¶^: Cases were staged according to the 1988 FIGO staging system. ^ζ^: Local recurrence after the date of initial surgical resection.

## Data Availability

The data in the paper can be found in the TCGA database (https://portal.gdc.cancer.gov/, accessed on 6 August 2023) and all data are publicly available.

## Supplementary Materials

The following supporting information can be downloaded at https://www.mdpi.com/2072-6694/15/16/4044/s1. Figure S1: Association of chemotherapy response status with patient age in the study cohort (median difference: 2.6 years). Figure S2: (a) Number of whole-slide images per class. (b) Distribution of the number of ROIs per slide. (c) Association of the number of ovarian cases with 5 ROIs per slide with chemotherapy response. There was no significant effect (Fisher’s exact *p* = 0.7906, odds ratio = 1.191). Figure S3: Effect of class imbalance on the network performance. Receiver operating characteristic (ROC) curves for the test set in the cases of (a) upsize and (b) downsize. Table S1: Association of chemotherapy response status with tumor grade in the study cohort (*p* = 0.3287, Fisher’s exact test). Table S2: Association of chemotherapy response status with tumor stage in the study cohort (*p* = 0.216, Fisher’s exact test). Table S3: Dataset information for chemo-resistant vs. chemo-sensitive classification (number of patients/WSIs, ROIs, and tiles in each category). Table S4: Multivariate analysis of overall survival for the 40-patient test set. Due to the small sample size and class imbalance, the stage and age variables do not show significant effects. The tests are underpowered. This table shows that histopathological score is an independent predictor of survival for the TCGA cohort. Table S5: Multivariate analysis of progression-free survival for the 40-patient test set. Due to the small sample size and class imbalance, the stage and age variables do not show significant effects. The tests are underpowered. This table shows that histopathological score is an independent predictor of progression-free survival for the TCGA cohort.
